# The Design, Characterizations, and Tumor Angiogenesis Inhibition of a Multi-Epitope Peptibody With bFGF/VEGFA

**DOI:** 10.3389/fonc.2020.01190

**Published:** 2020-07-17

**Authors:** Ligang Zhang, Yanrui Deng, Yinmei Zhang, Chunyan Liu, Simin Zhang, Wenhui Zhu, Yong Tang, Ning Deng

**Affiliations:** Department of Biology, Guangdong Province Engineering Research Center for Antibody Drug and Immunoassay, Jinan University, Guangzhou, China

**Keywords:** bFGF, VEGFA, Fc domain, peptibody, tumor angiogenesis

## Abstract

Tumor angiogenesis is dependent on growth factors, and inhibition of their pathways is one of the promising strategies in cancer therapy. However, resistance to single pathway has been a great concern in clinical trials so that it necessitates multiple targetable factors for developing tumor angiogenesis inhibitors. Moreover, the strategy of Fc fusion protein is an attractive platform for novel peptide agents, which gains increasing importance with FDA approval because of better immunogenicity and stability. Here, we applied the Fc fusion protein concept to bFGF/VEGFA pathways and designed a multi-epitope Peptibody with immunogenic peptides derived from human bFGF and VEGFA sequences. Immunization with Peptibody could elicit high-titer anti-bFGF and anti-VEGFA antibodies, activate T cells, and induce Th1/Th2-type cytokines. In *in vitro* experiments, the isolated anti-Peptibody antibody inhibited the proliferation and migration of A549 cells and human umbilical vein endothelial cells (HUVECs) by decreasing the MAPK/Akt/mTOR signal pathways. In the murine tumor model, pre-immunization with Peptibody suppressed the tumor growth and neovascularization of lung cancer by decreasing the production of bFGF/VEGFA/PDGF, the MAPK/Akt/mTOR signal pathways, and the activation of suppressive cells in tumor sites. Further, the biological characterizations of the recombinant Peptibody were investigated systematically, including protein primary structure, secondary structure, stability, and toxicity. Collectively, the results highlighted the strategy of bFGF/VEGFA pathways and Fc fusion protein in suppressing tumor progression and angiogenesis, which emphasized the potential of multiple targetable factors for producing enduring clinical responses in tumor patients.

## Introduction

The formation of blood vessels is critical not only for normal development but also for tumorigenesis and metastasis (1). Once solid tumors grow beyond a few millimeters, the angiogenic program is turned on to transport nutrients, oxygen, and metabolins, making tumor growth uncontrolled (2). This complex process requires proliferation, migration, and structural modification of endothelial cells, which are regulated by pro-angiogenic factors, such as basic fibroblast growth factor (bFGF) and vascular endothelial growth factor A (VEGFA) (3). Further, either alone or in combination, these two factors stimulate proteases and plasminogen activators in tumor tissues to degrade the basement membrane, which promotes tumor metastasis and endothelial cells recruitment for neovascularization (4). In addition, bFGF and VEGFA can synchronize platelet-derived growth factor (PDGF) and its receptor synergistically to facilitate blood vessel formation by modulating their expression and activation (5). Aberrant expression of bFGF and VEGFA are implicated in a broad range of solid tumors (6–8). These endogenous growth factors work as primary regulators in tumor progression and angiogenesis through autocrine and paracrine activation of their cognate receptors (9). Since solid tumor is highly vascularized, the strategy of anti-angiogenesis is more attractive. bFGF and VEGFA have been become the popular targetable genes with FDA approval, such as the inhibition of growth factors, receptors, and intracellular kinases (10–15). Nonetheless, resistance to single pathway often occurs in the presence of activated alternative growth factors in clinical therapy, followed by a compensatory restoration of tumor growth (16). In order to produce enduring clinical responses in cancer patients, the strategy targeting multiple factors might be a feasible improvement.

Fc fusion protein, in which Fc domain of IgG isotypes is joined to recombinant protein, is considered as a promising platform for novel peptide agents (17). Drugs derived from peptide often suffer from short serum half-life owing to their low molecular mass and fast renal clearance (18). In contrast, Fc fusion protein generated from the genetic linkage of effector moiety (cytokines or antibody fragments) and Fc domain (human IgG1) is believed to be effective in human therapy, as exemplified by Etanercept (Enbrel), a TNFR2-Fc fusion protein that reduces TNF in rheumatoid arthritis (RA) (19). Indeed, it can induce potent physiological responses through the interaction with Fc receptor. The binding of Fc domain and neonatal Fc receptor (FcRn) expressed in epithelial, endothelial, and leukocyte cells protects the effector protein from lysosomal breakdown, increasing the half-life and therapeutic activity (20). Abatacept (Orencia), a CTLA-4-Fc fusion protein that abrogates T cell activation in RA, has a half-life of more than 10 days (21). The binding capability to Fc gamma receptor (FcγR) family can trigger certain Fc-mediated effector functions, such as complement-dependent cytotoxicity, antibody-dependent cell-mediated cytotoxicity, and modulations of other immune cells (22). Other properties such as solubility and stability have considerable improvements with Fc domain (23). Additionally, this technology facilitates the downstream purification, allowing the use of Protein A chromatography, with high affinity to Fc domain (24). Aflibercept (Eylea and Zaltrap) is a soluble recombinant Fc fusion protein containing extracellular domains of VEGFR1 and VEGFR2 (12). Consequently, Fc fusion protein is now well-established as therapeutics with FDA approval, and such strategy for novel peptide agents will gain increasing importance in cancer therapy (25). However, Fc domain is also a foreign antigen, so the immunogenicity of Fc domain in the Fc fusion protein should be included.

In this study, we applied the Fc fusion protein concept to both bFGF and VEGFA pathways and investigated the contribution of this anti-angiogenesis strategy in tumor therapy. The recombinant Fc fusion protein (Peptibody) we designed was composed of three human immunogenic bFGF peptides, three human immunogenic VEGFA peptides, and a human IgG1 Fc domain, which were derived from bioinformatic prediction and phage display. Above all, the immunogenicity of Peptibody should be evaluated systematically in mice, including whether it could elicit specific humoral and cellular immune responses and the activation of relevant cytokines. Next, we examined the inhibitory effects and mechanisms of Peptibody on tumor progression and angiogenesis, using lung cancer cell line A549 and vascular cell line HUVECs (human umbilical vein endothelial cells) *in vitro* experiments and murine tumor model of Lewis lung cancer (LL-2). Further, we enhanced our understanding of detailed biological characterizations of the recombinant Peptibody, including protein primary structure, secondary structure, stability, and toxicity. We hoped that the strategy of multiple targetable factors and Fc fusion protein would provide a broad-acting therapeutic modality for tumor angiogenesis inhibition.

## Materials and Methods

### Construction of pET-28a-bFGF/VEGFA-Fc Plasmid and the Expression and Purification Tests

The immunogenic peptides of human bFGF and VEGFA were obtained from a phage peptide library scanning and bioinformatic analysis according to the prediction by Saha et al. and El-Manzalawy et al. (26–28). The oligonucleotide fragments of bFGF/VEGFA-Fc (human IgG1) with linkers were synthesized by Sangon Biotech (Shanghai, China) and inserted into the vector pET-28a by restriction enzymes *Nhe*l, *Bam*HI, and *Xho*l, creating pET-28a-bFGF/VEGFA-Fc (pET-28a-Peptibody). After validation by restriction enzymes and PCR assays, the recombinant plasmid was expressed in *E. coli* BL21 (DE3) and induced with 0.1 mM IPTG in the mid-log phase at 28°C. The recombinant Peptibody was purified by gradient NaCl-PB solution using cation-exchange and hydrophobic chromatography. The peptide candidates and primers were presented in Table S1.

### Cell Culture

Human lung cancer cells A549, HUVECs, and murine Lewis lung cancer cells LL-2 were available in our laboratory. Cells were cultured in DMEM (Gibco, Langley, OK, USA) supplemented with 10% fetal bovine serum (FBS, Gibco), 100 U/ml penicillin (Gibco), and 100 μg/ml streptomycin (Gibco) at 37°C in a humidified atmosphere of 5% CO_2_. If necessary, cells were activated with 10 ng/ml bFGF.

### Mice and Immunization

The BALB/c and C57BL/6 mice (female, 6 weeks) were purchased from the Experimental Animals Center of Southern Medical University in Guangzhou, China. The mice were housed in specific pathogen-free environment and the treatment of animals was approved by the Institutional Animals Care and Use Committee on animal research in Jinan University, Guangzhou, China. Every 2 weeks, the mice were injected subcutaneously (s.c.) with Peptibody (100 μg/mouse), the recombinant Fc domain (100 μg/mouse), and the same volume of PBS for three times, respectively. Four weeks later, mice were sacrificed and organs and blood were extracted.

### Enzyme-Linked Immunosorbent Assay (ELISA)

The human bFGF (#P09038, R&D Systems, Minneapolis, MN, USA) and VEGFA (#AAA36804, R&D Systems) were dispensed into 96-well plates (50 ng/well, overnight, 4°C). After 5% nonfat milk blocking (1 h), the plates were incubated with serially diluted sera from Peptibody and PBS-immunized mice. After 45-min incubation (37°C) of HRP-conjugated goat anti-mouse IgG (1:2000, #D110087, Sangon Biotech, Shanghai, China), the absorbance at 450 nm was read by a microplate reader (BioTek Instruments, Winooski, VT, USA). The antibody titers were defined as the reciprocal of serum dilution. PBS and the recombinant Fc domain served as the control. The antibody subtypes were measured by Isotyping ELISA Kit (#SEK003, Sino, Beijing, China). The expression levels of IFN-γ and IL-2/4/6 in the spleen and serum were determined by pre-coated plates ELISA Kit (#430808, #431008, #431108, #431308, BioLegend, San Diego, CA, USA). The expression level of histamine in the serum and the binding activity of Peptibody were detected by double-antibody sandwich-ELISA (ds-ELISA).

### Flow Cytometry (FCM)

For T cell analysis, the splenocytes (5 × 10^5^/well) were incubated with PE-labeled anti-mouse CD4 (#100407, BioLegend) and Percp-labeled anti-mouse CD8 (#100731, BioLegend) antibodies. For cell cycle analysis, A549 cells (1 × 10^5^/well) were incubated with 200 μg/ml anti-Peptibody antibody, fixed with 70% ethanol, and stained with PI. Irrelevant IgG, anti-Fc antibody, and anti-full-length bFGF antibody served as the control. The labeled splenocytes and stained A549 cells were detected by FACSCalibur flow cytometer (BD Biosciences, CA, USA). T cells were calculated by FlowJo software (FlowJo LLC, OR, USA) and cell cycle distribution was analyzed by ModFit LT software (Verity Software House, ME, USA).

### Cell Viability

A549 cells and HUVECs (1 × 10^3^/well) were seeded into 96-well plates and anti-Peptibody antibody was added at increasing concentrations, from 25 to 400 μg/ml. Cells were cultured for a further 72 h and cell viability was determined using CCK-8 kit (10 μl, #CK04, Dojindo, Kumamoto, Japan). The absorbance at 450 nm was read by a microplate reader. Irrelevant IgG, anti-Fc antibody, and anti-full-length bFGF antibody served as the control.

### Western Blotting

Cells were lysed with RIPA buffer (#P0013, Beyotime, Jiangsu, China) containing protease and phosphatase inhibitors. Protein concentrations were measured by BCA kit (Thermo Scientific, San Jose, CA, USA). Each sample of 20 μg protein was separated on 10% SDS-PAGE gels and blotted onto PVDF membranes (#IPVH00010, Millipore, Bedford, MA, USA). Primary antibodies used were anti-mTOR (1:1000, #2983), anti-Akt (1:1000, #4691), anti-p-Akt (Ser473, 1:2000, #4060), anti-MAPK (1:1000, #4695), anti-p-MAPK (Thr202/Tyr204, 1:2000, #4370), and anti-GAPDH (1:1000, #5174) (Cell Signaling Technology, Danvers, MA, USA); anti-VEGFA (1:10,000, #ab52917, Abcam, Cambridge, UK); and anti-His (1:1000, #D110002, BBI Life Sciences, Shanghai, China). Secondary antibody used was HRP-conjugated goat anti-rabbit IgG (1:1000, #7074, Cell Signaling Technology). Immunoreactivity detection was performed using super ECL plus (#WBKLS0100, Millipore) and Gel Documentation System (Bio-Rad, Hercules, CA, USA). GAPDH served as loading control and the signal intensities were quantified by ImageJ software (NIH, Bethesda, MD, USA).

### Wound-Healing Assay

Cells (3 × 10^5^ cells/well) were seeded in 6-well plates and incubated with 200 μg/ml anti-Peptibody antibody for a further 24 h. The monolayer cells were scraped in a straight line and washed. Photographs of the scratches were taken at 0, 12, and 24 h using an inverted microscope (Olympus, Tokyo, Japan). The area without cells of the defined site along each scratch was measured by ImageJ software and given an average of all measurements. Irrelevant IgG, anti-Fc antibody, and anti-full-length bFGF antibody served as the control.

### Matrigel Invasion Assay

Cells (2 × 10^5^ cells/well) suspended in 100 μl of basal medium were seeded into the upper transwell chambers (#353097, BD Bioscience, San Jose, CA, USA) coated with Matrigel (#356234, BD Bioscience), and 700 μl of medium containing 10% FBS was plated into the bottom. After incubating with 200 μg/ml anti-Peptibody antibody for 24 h, the cells were fixed with 4% paraformaldehyde and stained with 0.1% crystal violet. The cells on the surface of upper chamber were removed. The migrated cells were photographed by inverted microscope and counted in five random fields. Irrelevant IgG, anti-Fc antibody, and anti-full-length bFGF antibody served as the control.

### Mouse Model and Survival Study With LL-2 Cells

As described above, the C57BL/6 mice (*n* = 7) were immunized with Peptibody, human full-length bFGF (R&D Systems) as a positive control and PBS as a negative control. Four weeks later, mice were inoculated with LL-2 cells (2 × 10^6^/mouse) under the left front flank. Tumor growth was measured by a caliper and tumor volume was calculated using the formula: Volume = *a* × *b*^2^/2 (*a*, the longer diameter; *b*, the shorter one). After sacrifice, tumors were stripped and weighed. Animal survival was determined on the basis of tumor sizes reaching the longest diameters allowable (20 mm). To assess the effects of Peptibody on tumor growth, the tumor volumes at different time points were subjected to mixed-effects models for repeated-measures ANOVA.

### Immunofluorescence (IF) and Hematoxylin–Eosin (HE) Staining

Tumor tissues from the mouse model were fixed in 4% paraformaldehyde and embedded in paraffin. After deparaffinization, the sections were incubated with 10 mM sodium citrate buffer (pH 6.0) and 3% H2O2 to repress the endogenous peroxidase activity, followed by 5% BSA and 0.05% Triton X-100 blocking treatment. For IF assay, primary antibodies used were anti-CD31 (1:20, #ab28364), anti-LYVE-1 (5 μg/ml, #ab14917), anti-bFGF (1:200, #ab8880), and anti-VEGFA (1:250) (Abcam); anti-PDGF (1:200, #GB11261), anti-IL-10 (1:200, #GB11108), and anti-TGF-β (1:200, #GB14152) (Servicebio, Wuhan, China); anti-mTOR (1:200), anti-p-Akt (1:400), anti-p-MAPK (1:200), and anti-CD11b (1:800, #17-0112-8, eBioscience, San Diego, CA, USA); and anti-EGF (1:200, #sc-374255, Santa Cruz Biotechnology, Santa Cruz, CA, USA). Cell nuclei were visualized with DAPI (5 ng/ml, Invitrogen, New York, NY, USA) and fluorescence was collected by a fluorescence microscope (Olympus). For HE staining, the sections were stained with HE, and the images were captured by an inverted microscope.

### Liquid Chromatography–Mass Spectrometry (LC-MS)

The mass spectrometer used was Q Exactive (Thermo Scientific). For sequencing and peptide mapping, the data were processed by BiopharmaLynx 1.3 software. For molecular weight (MW), the data were calculated through deconvolution by ProMass for XcaliburTM software.

### Circular Dichroism (CD)

Using Chirascan Plus V100 spectrometer (Applied Photophysics, Leatherhead, Surrey, UK), the CD spectra of Peptibody were recorded in a cylindrical quartz cuvette at room temperature. The recorded spectra were analyzed by Pro-Data Viewer in the model of Milli-Degress.

### Tm and Tagg

OPTIM instrument (Unchained Labs, San Francisco, CA, USA) was used to detect the thermal unfolding transition mid-point temperature (Tm) and aggregation onset temperature (Tagg). The linear ramp of temperature (15–95°C) was increased at 10°C/min. The intrinsic tryptophane fluorescence and static light scattering (SLS) at 266 and 475 nm were calculated and plotted.

### Statistical Analysis

The experiments were repeated three times at least and the data were presented as mean ± standard deviation (SD, error bars). The statistical significance of differences between experimental groups was analyzed by SPSS 19.0 software and Student's *t*-test. *P* < 0.05 was considered to be statistically significant.

## Results

### Design of the Recombinant Peptibody and the Expression and Purification Tests

Six peptide candidates targeting B cell and T cell epitopes were selected to construct the recombinant Peptibody fusion protein with human IgG1 Fc domain (Table S1). Three bFGF epitope peptides were used: AMKEDGRLLASK (75–86, b1), IHPDGRVDGVREKS (34–47, b2), and RLESNNYNTYRSRKYTS (97–113, b3). The three VEGFA epitope peptides used were QKRKRKKSRYKS (331–342, V1), RPKKDRARQ EKKS (311–323, V2), and VASAVFYSALVE (phage peptide library, V3). The synthesized sequences bFGF/VEGFA-Fc were inserted into pET-28a by restrictions enzymes *Nhe*l, *Bam*HI, and *Xho*l (Figure 1A). The expression vector pET-28a-Peptibody was identified by restriction digestion and transformed into *E. coli* BL21 (DE3). The Peptibody strains were induced with 0.1 mM IPTG (Figure 1B). The target protein was purified by gradient NaCl-PB solution using cation-exchange and hydrophobic chromatography (Figure 1C).

**Figure 1:** Schematic representation of the recombinant pET28a-Peptibody and the expression and purification tests. **(A)** The synthesized sequences of bFGF/VEGFA and Fc domain with linkers were inserted into pET28a by restriction enzymes *Nhe*l, *Bam*HI, and *Xho*l. (a) Construction of the prokaryotic expression vector. (b) Combination diagram of the peptide candidates and linkers. **(B)** Identification of the recombinant vector and expression of Peptibody. (a) Agarose gel of restriction digestion and PCR assays. Lanes 1 and 2, digestion and PCR product of bFGF/VEGFA and Fc domain. M, DNA ladder marker. (b) SDS-PAGE and Western blotting assays. Lanes 1 and 2 and 7 and 8, induction sample. Lanes 3 and 5, non-induction sample. Lanes 4 and 6, empty vector sample. The primary antibody was monoclonal anti-human VEGFA of rabbit. M, MW marker. **(C)** The purification procedures of Peptibody. (a) Cation-exchange chromatography. Lanes from left to right, load sample, FT, 0.5 M NaCl-PB, 0.7 M NaCl-PB, 1 M NaCl-PB, and 0.5 M NaOH. (b) Hydrophobic chromatography. Lanes from left to right, load sample, FT, 2 M NaCl-PB, 1 M NaCl-PB, 0.6 M NaCl-PB, 20 mM PB, ddH_2_O, and the purified product. FT, flow through; M, MW marker. The target protein was 37.4 kDa in which the red arrow pointed at.

### Peptibody Elicited Superior Immune Responses in Mice

The BALB/c mice were injected s.c. with Peptibody (100 μg/mouse), the recombinant Fc domain (100 μg/mouse), and PBS, respectively. After sacrifice, blood was extracted and the antibodies were purified by Protein G affinity chromatography (Figure 2A). To identify the immune signatures of Peptibody, the sera and spleens were collected to analyze the antibody titers, T cell activation, and relevant cytokines. The titers of anti-bFGF, anti-VEGFA, and anti-Fc antibodies were about 1:16,000, 1:2000, and 1:4000, respectively, while most of the antibody subtypes were IgG (Figures 2B,C). The proportions of CD4^+^ T and CD8^+^ T cells were increased by 10.28 ± 1.16% and 5.32 ± 0.91% (Figure 2D). Further, the Th1/Th2 cell-related cytokines including IFN-γ and IL-2/4/6 were obviously up-regulated (Figure 2E). As a foreign antigen, immunization with Fc domain alone could also activate some immune responses, but the signatures were weaker than Peptibody (Figures 2B,D). Collectively, Peptibody showed superior immune signatures including specific B cell and T cell responses and relevant cytokine activation, which might be used as a potential agent for tumor treatment.

**Figure 2:** Immunogenicity of Peptibody fusion protein. **(A–E)** The BALB/c mice were injected three times s.c. with Peptibody (100 μg/mouse). Four weeks later, mice were sacrificed and blood was extracted. PBS and the recombinant Fc domain served as the control. **(A)** The purification of anti-Peptibody antibody by Protein G affinity chromatography. Lanes from left to right, sera, FT, 100 mM glycine (gly, pH 3.6), and non-reducing and reducing antibodies. **(B)** The antibody titers were detected by ELISA assay. (a) Anti-bFGF/VEGFA and anti-Fc antibodies. (b) Anti-Fc antibody. **(C)** The subtypes of anti-Peptibody antibody were detected by ELISA assays. **(D)** Cells were stained with PE-labeled anti-mouse CD4 and Percp-labeled anti-mouse CD8 antibodies. CD4^+^ T and CD8^+^ T cells were analyzed by Flowjo software. **(E)** The activation of IFN-γ and IL-2/4/6 were detected by ELISA assay. (a–d) Cytokines in the spleen. (e–g) Cytokines in the sera. *p < 0.05, ***p < 0.001, ****p < 0.0001.

### Anti-Peptibody Antibody Inhibited the Proliferation, Migration, and Invasion of A549 Cells and HUVECs

To investigate the inhibitory effects of anti-Peptibody antibody on tumorigenesis and angiogenesis, assays of CCK-8, signal pathway, cell cycle, wound healing, and Matrigel invasion were conducted *in vitro*. The results showed that the proliferation of A549 cells and HUVECs was obviously suppressed in a dose-dependent manner, with inhibition rates of 65.74 ± 2.95% and 24.17 ± 8.45% at 400 μg/ml (Figure 3A, Figure S1A). The MAPK/Akt/mTOR signal pathways were down-regulated in a dose- and time-dependent manner (Figure 3B, Figure S1B). The DNA replication of A549 cells was inhibited and cell cycle was arrested at the G1 phase (Figure 3C). The migration and invasion of A549 cells and HUVECs were obviously inhibited, with inhibition rates over 60% (Figures 3D–F, Figures S1C,D). Moreover, the irrelevant IgG and anti-Fc antibody did not show any inhibitory effects while the inhibition of anti-Peptibody antibody was stronger than the positive control anti-full-length bFGF antibody. The results suggested that the anti-Peptibody antibody could inhibit the progression of tumor and vascular endothelial cells *in vitro*.

**Figure 3:** Inhibitory effects of anti-Peptibody antibody on the proliferation, migration, and invasion of A549 cells. **(C–E)** A549 cells were treated with 200 μg/ml antibodies for 24 h. (a) Irrelevant IgG. (b) Anti-Fc. (c) Anti-Peptibody. (d) Anti-full-length bFGF. **(A)** A549 cells were treated with increasing concentration of antibodies, and cell viability was determined by CCK-8 assay. **(B)** MAPK, Akt, and mTOR expression and/or activation were evaluated in A549 cells treated with anti-Peptibody antibody. (a) In a dose-dependent manner. (b) In a time-dependent manner. Expression levels of MAPK, Akt, mTOR, and GAPDH were detected, respectively. Phosphorylation of MAPK and Akt (p-MAPK and p-Akt) was detected, as indicated. GAPDH served as loading control. Total proteins of each sample (20 μg) were analyzed by SDS-PAGE. **(C)** Cells were stained with PI and cell cycle phase distribution was analyzed by ModiFit software. **(D)** The effect of anti-Peptibody antibody on A549 cell migration was measured by wound-healing assay. Representative images showed the scratched areas of A549 cells. **(E)** The effect of the anti-Peptibody antibody on A549 cell invasion was measured by transwell chamber assay. Representative images showed the invaded A549 cells. **(F)** (a, b) Statistical analysis of A549 cell migration and invasion data. Scale bars, D: 100 μm, E: 50 μm. **p < 0.01.

### Peptibody Inhibited the Tumor Growth and Angiogenesis of Lung Cancer and Promoted Survival in Mice

The C57BL/6 mice (*n* = 7) were pre-immunized with Peptibody and LL-2 cells (2 × 10^6^/mouse) were inoculated under the left front flank. Tumor growth of the challenged mice was suppressed by 77.31% and the life span was prolonged by 12 days, with a median survival time of 33 days (Figure 4A). The generation of microvessels and lymph vessels was decreased by 49.83 and 69.31%, respectively (Figure 4B). The lung cancer markers in the serum including AFP, NSE, FER, CA50, CA125, CA153, and CA199 were in the range of threshold permitted, which means that the tumor metastasis did not occur (Table S2). In the tumor tissues, the expression levels of bFGF, VEGFA, and PDGF were down-regulated owing to Peptibody immunization (Figure 4C). Activation of the MAPK/Akt/mTOR signal pathways and the MDSCs/TAMs-related cytokines in TME were obviously blocked, including IL-10, TGF-β, EGF, and VEGFA (Figure 5). All the inhibitory effects of Peptibody were stronger than the positive control, full-length bFGF. The results suggested that Peptibody could significantly suppress the tumor growth and angiogenesis of lung cancer through blockade of the MAPK/Akt/mTOR signal pathways and suppressive cells in TME. Without alternative activation, the life span of the challenged mice was well-improved.

**Figure 4:** Inhibitory effects of Peptibody on the tumor growth and angiogenesis in mice and the survival promotion. **(A**–**C)** C57BL/6 mice (*n* = 7) were s.c. given injection of Peptibody (100 μg/mouse), human full-length bFGF (100 μg/mouse), and the same volume of PBS for three times, respectively. Four weeks later, LL-2 cells (2 × 10^6^/mouse) were inoculated under the left front flank. **(A)** (a) Tumor images. (b) Tumor volume. (c) Tumor weight. (d) Survival time. **(B,C)** IF staining of microvessels, lymph vessels, and angiogenic factors of the stripped tumors. Left panel, representative images. Right panel, statistical analysis of data. Scale bars, B: 100 μm, C: 100 μm. *p < 0.05.

**Figure 5:** Inhibitory effects of Peptibody on the MAPK/Akt/mTOR signal pathways and suppressive cells in the stripped tumors. Phosphorylation of MAPK and Akt (p-MAPK and p-Akt) and expression levels of mTOR, CD11b, IL-10, TGF-β, and EGF of the stripped tumors were detected by IF staining. Left panel, representative images. Right panel, statistical analysis of data. Scale bars, 100 μm. *p < 0.05, **p < 0.01.

### Primary Structure Determination of Peptibody by Sequencing and Peptide-Mapping Analysis

For recombinant protein, the composition of N-terminal, C-terminal, and peptide mapping, which is closely related to biological functions, should be totally certified, using Edman degradation and LC-MS. Peptibody was treated with six proteolytic enzymes (trypsin, chymotrypsin, Asp-N, Glu-C, Lys-C, and Lys-N) and digested into amenable peptide fragments for LC-MS analysis. The results showed that the 15 amino acids of N-terminal were Met-Gln-Lys-Arg-Lys-Arg-Lys- Lys-Ser-Arg-Tyr-Lys-Ser-Gly-Gly (Figure S2) and that of C-terminal was Lys (K, Table S3), the same as the theoretical sequence. With more proteases, the whole sequence was detected at the coverage of trypsin 87.5%, chymotrypsin 75.3%, and Glu-C 76.7% (Table S4). The peptide mapping was shown in Figure S3 and Table S5, which could be used as a valuable standard to certify the complete expression and primary structure of Peptibody (29). The pI and MW were 8.93 and 37.415 kDa, within the errors allowed (Figures S4A,B). The binding specificity after production was analyzed using anti-VEGFA and anti-His antibodies (Figure S4C).

### Secondary Structure Determination of Peptibody by CD Scanning

CD instrument has become a valuable technique to estimate the structure of unknown protein specially in the solution. Structures of various types give rise to a characteristic shape and magnitude of CD spectra (30). The secondary structure composition was estimated by CD scanning to further understand the Peptibody biological immunogenicity. The data confirmed the presence of alpha helix (9.0%), anti-parallel (31.3%), parallel (5.4%), beta sheet (22.2%), and random coil (39.1%) in the secondary structure, indicating a better immunogenicity of Peptibody (Figure 6A and Table S6).

**Figure 6:** CD spectroscopy and thermostability analysis of Peptibody. **(A)** CD scanning spectra of the far and near UV. (a, b) The absorbance and CD spectra of sample in the far UV. (c, d) The absorbance and CD spectra of sample in the near UV. (e) The CD spectra of standard in the far and near UV. (f) The predicted secondary structure of Peptibody. **(B)** The thermostability of Peptibody was detected by temperature ramp assay. (a) Intrinsic tryptophane fluorescence. (b) SLS at 266 nm.

### Assessing the Stability of Peptibody

For thermostability, the Tm and Tagg of Peptibody were simultaneously determined by OPTIM instrument. The fluorescence intensity from tryptophane and SLS will be strengthened if proteins unfold and aggregate with temperature going up. The data confirmed the presence of four Tm (33.5 ± 0.44, 49.7 ± 0.86, 71.3 ± 0.38, and 80.9 ± 1.80°C) and one Tagg (69.2 ± 0.47°C), which means that Peptibody started to unfold at 33.5 ± 0.44°C, aggregate at 69.2 ± 0.47°C, and totally degraded at the temperature over 90°C (Figure 6B and Table S7). The substantial thermostability of Peptibody could bring convenience to its preparation research in the following SDS-PAGE, Western blotting, and ds-ELISA assays. The samples and binding activity started to break down at the temperature over 37°C, pH below 4 or over 9. As for buffer and stabilizer, Tris–HCl and sucrose were unsuitable (Figure S5). The results suggested that Peptibody could be produced at room temperature (<28°C) but at least stored at 4°C. The buffer was normal saline (NS, pH 7.4) for human use but the stabilizer and expiration time of Peptibody needed further examinations.

### Assessing the Toxicity of Peptibody

As for agents from gene engineering, most of the costs are sunk into failures owing to safety findings. Thus, the safety and side effects of Peptibody should be systemically evaluated (31). The regular observation and blood of the Peptibody-immunized mice were collected. The organs including heart, liver, spleen, lung, kidney, hystera, and spermary were analyzed by HE staining. The results showed that no differences of feeding, water drinking, and body weight were found compared with the control (Figure S6A). The blood routines were in the range of threshold permitted (Table S8). Additionally, histamine, an indicator to allergy, was maintained at a low level (Figure S6B). The cell morphology of each organ was healthy and no inflammatory cell infiltration was observed (Figure S7). Therefore, Peptibody had little pathological side effects in mice, but its safety was essential for further observation. These findings might provide pre-clinical evidence to support the potential application of Peptibody in cancer therapy.

## Discussion

For peptide candidates of Peptibody, the antigenic index and secondary structure were crucial in the prediction. We selected B cells and T cell epitopes of human bFGF/VEGFA, and in CD scanning, the epitopes were abundant in alpha helix, anti-parallel, parallel, beta sheet, and random coil. The effector peptides fused with Fc domain are highly immunogenic to induce immune responses, relative to native antigens (32). The Peptibody we designed could elicit high-titer anti-bFGF/VEGFA antibodies, T cells, and Th1/Th2-type cytokine activation in mice, suggesting that it could stimulate specific humoral and cellular immune responses. Meanwhile, it was possible that the immune responses to Peptibody might be dependent on the sequence differences between human and mice. If so, the Peptibody fusion protein can be recognized as foreign antigens and induce antibodies in mice, but may be recognized as self-antigen in human. To rule out this suspicion, clinical trials are needed. According to NCBI matching, the epitopes we selected are so similar to murine bFGF/VEGFA, only one to three different amino acids, that it is expected to elicit dramatic immune responses in human body when it occurs in mice. In case of failure, the fusion protein targeting both bFGF/VEGFA is still promising, because, in turn, we can use peptide candidates of other species to elicit immune responses in clinical trials.

Lung cancer, full of neovascularization, is the most commonly diagnosed cancer with the highest mortality rate (33). bFGF and VEGFA were highly expressed in A549 and LL-2 cells (34, 35). Consequently, the tumor growth and angiogenesis of lung cancer were obviously suppressed by Peptibody immunization. It has been reported that the expression levels of PDGF and bFGF will be increased in the patients with long-term use of Bevacizumab, followed by a compensatory restoration of angiogenesis (36). In the mice immunized with full-length bFGF alone, VEGFA was up-regulated compared with PBS immunization while PDGF was up-regulated compared with Peptibody immunization. The expression levels of bFGF and VEGFA were reduced and we did not see alternative activation of PDGF in the tumor sites immunized with Peptibody (Figure 4C). It is necessary that alternative activation of any other related angiogenic factors should be identified in the following experiments. Therefore, the strategy targeting both bFGF and VEGFA signal pathways may help strengthen the therapeutic efficacy of tumor patients and relieve the resistance (37).

We believe that the mouse anti-human bFGF/VEGFA antibodies elicited by Peptibody can neutralize the dissociative murine bFGF/VEGFA in tumor microenvironment (TME) and the pathways related in the tumor cells will be down-regulated, resulting in tumorigenesis and angiogenesis inhibition. The anti-Peptibody antibodies isolated from the serum were polyclonal antibodies, including anti-bFGF/VEGFA and Fc antibodies. Although immunization with the recombinant Fc domain alone could also activate some immune responses in mice, the anti-Fc antibody did not show any inhibitory effects on tumor progression and angiogenesis *in vitro*. Thus, the inhibitory effects were more specific due to antibodies against the bFGF/VEGFA epitopes we designed. However, the anti-bFGF/VEGFA antibodies may or may not be against all the six peptide candidates and some of them may not work. We are not sure which epitopes are responsible for the inhibitory effects. Hence, we are planning to immunize the epitopes independently so that we can figure out the specific epitopes and improve the fusion protein.

Activation of FGFR and VEGFR can trigger downstream MAPK/Akt signal pathways, which play key roles in the behaviors of tumor and endothelial cells including proliferation, survival, and motility (38, 39). Moreover, the Akt signal pathway positively regulates mTOR, which has been associated with bad prognosis and earlier recurrence in tumor treatment (40). In particular, the mTOR inhibitor rapamycin has showed potent anti-tumor effects (41). The activation of MAPK/Akt/mTOR signal pathways were simultaneously down-regulated when treated with anti-Peptibody antibody in A549 cells, HUVECs, and Peptibody in LL-2-bearing mice. The cellular events of tumor and endothelial cells were suppressed, following tumorigenesis and neovascularization depression. However, our knowledge about the inhibition is still very limited, especially regarding the mechanism of down-regulating downstream signal pathways and gene expression for tumorigenesis and angiogenesis.

Although immunotherapeutic approaches have been approved in several tumors, the anti-tumor efficacy appears to be modest in clinical therapy (42). This tumor resistance might be partly related to the highly immunosuppressive TME (43). The immunoregulatory mechanisms responsible for tumor escape have been identified and what we pay the most attention to is the activation of suppressive cells including myeloid-derived suppressor cells (MDSCs) and tumor-associated macrophages (TAMs) (44, 45). VEGFA and other factors activate MDSCs (Gr-1^+^ CD11b^+^) to suppress host immune responses, enhance angiogenesis, and promote tumorigenesis through secretion of versatile immunosuppressive factors, such as IL-10 and TGF-β (46). The IL-4-activated TAMs (M2 phenotype, CD11b^+^ CD11c^−^) enhance the malignancy of tumor cells by releasing a variety of cytokines, including EGF and VEGFA (47). With Peptibody immunization, the CD11b^+^ cells and related cytokines of suppressive cells were obviously down-regulated, suggesting that Peptibody could destroy the immunosuppressive TME and produce dramatic inhibitory effects on tumor growth and angiogenesis.

The recombinant protein fused with Fc domain conferred certain advantages to stability. Peptibody occurred to degrade and aggregate at higher temperature, which would cut the costs for production, transportation, and storage. Moreover, Peptibody exhibited favorable stability in common buffers and stabilizers, expecting a longer half-life and a better efficacy. Fortunately, little side effects of organs, allergy, and survival were detected, but more toxicity examinations should be performed, such as the inhibitory effects of Peptibody on normal wound healing and other toxicity evaluation.

## Conclusions

In conclusion, this study developed a multi-epitope Peptibody with bFGF/VEGFA, which consisted of three human bFGF peptides and three human VEGFA peptides with human IgG1 Fc domain. Immunization with Peptibody could induce high-titer anti-bFGF/VEGFA antibodies, activate T cells, and induce Th1/Th2 type cytokines. The anti-Peptibody antibody inhibited the proliferation and migration of A549 cells and HUVECs by decreasing the MAPK/Akt/mTOR signal pathways. In murine model, pre-immunization with Peptibody suppressed tumor growth and angiogenesis to promote survival time. Additionally, the primary and secondary structures of Peptibody were systematically detected. With satisfactory stability and toxicity, the Peptibody fusion protein targeting both bFGF and VEGFA may provide a broad-acting therapeutic modality for tumor angiogenesis.

## Data Availability Statement

The datasets presented in this study can be found in online repositories. The names of the repository/repositories and accession number(s) can be found below: FigShare, https://doi.org/10.6084/m9.figshare.12444770.v1.

## Ethics Statement

The animal study was reviewed and approved by Institutional Animals Care and Use Committee on animal research in Jinan University, Guangzhou, China.

## Author Contributions

LZ and YD designed and performed the experiments and drafted the manuscript. YZ, CL, SZ, and WZ participated in the experiments. ND and YT supervised this study. All authors read and approved the final manuscript.

## Conflict of Interest

The authors declare that the research was conducted in the absence of any commercial or financial relationships that could be construed as a potential conflict of interest.
